The article "miR-193a-5p Enhances the Radioresistance of Pancreatic Cancer Cells by Targeting ZFP57 and Activating the Wnt Pathway" was published in 2022. Journal: J Oncol.

# miR-193a-5p Enhances the Radioresistance of Pancreatic Cancer Cells by Targeting ZFP57 and Activating the Wnt Pathway

**DOI:** 10.1155/2022/8071343

**Published:** 2022-10-14

**Authors:** Lulu Tan, Zhihua Chen

**Affiliations:** ^1^Department of Radiation Oncology, Hainan General Hospital, Hainan Affiliated Hospital of Hainan Medical University, Haikou, Hainan, China; ^2^Department of Digestive Medicine, Haikou People's Hospital, Haikou, Hainan, China

## Abstract

This study was to investigate whether miR-193a-5p and ZFP57 are involved in the radioresistance of pancreatic cancer and to explore its working mechanism. Pancreatic cancer tissues were harvested from patients who achieved CR (complete remission) and PR (partial remission) and those who achieved PD (progressive disease) and SD (stable disease). The mRNA and protein expressions of ZFP57 and miR-193a-5p were determined by RT-qPCR and WB (Western blot), respectively. For *in vitro* experiments, the parental BxPC-3 cell line was irradiated by X-ray at a total dose of 40 Gy to induce the irradiation-resistant subtype BxPC-3-RR. ZFP57 was downregulated in radioresistant pancreatic cancer cells. The results of dual-luciferase reporter gene assay, RNA pull-down assay, RT-qPCR, and WB confirmed that miR-193a-5p targeted ZFP57 and inhibited ZFP57 expression. The MTT assay and the colony formation assay showed that the radioresistant pancreatic cancer cells had higher viability and survival fraction. The results of WB indicated that in the radioresistant pancreatic cancer cells, the cyclin D1, Bax, CDk4, cleaved caspase-3, Bcl-2, and *γ*-H2AX proteins were upregulated to varying degrees. The results of the *in vitro* nude mouse experiment were consistent with those of *in vivo* experiments. According to the cell transfection and salvage experiments, miR-193a-5p down regulated ZFP57 after radiotherapy. As a result, the Wnt pathway was activated, which further induced radioresistance of pancreatic cancer cells. Our experiments showed that the miR-193a-5p/ZFP57/Wnt pathway mediated the radioresistance of pancreatic cancer cells, providing novel clues for the treatment of pancreatic cancer.

## 1. Introduction

Pancreatic cancer is a common malignancy featured by a low early discovery rate and a notoriously high malignancy. At present, the overall 5-year survival rate of pancreatic cancer is only 2%-9% [1]. Due to metastases of pancreatic cancer even at an early stage, only 10%-15% of pancreatic cancer patients have the opportunity to receive surgery after diagnosis. Even for those who have been surgically treated, the outcomes are limited due to high postoperative recurrence and metastasis rates. Radiotherapy, together with chemotherapy, is indicated for nearly all pancreatic cancer patients with a benefit in overall survival (OS), especially in those patient with metastasis [2, 3]. Radioresistance is the primary obstacle for better outcomes of radiotherapy. Identification of specific targets of radioresistance and regulation of these targets are expected to enhance the radiosensitivity of pancreatic cancer and improve the therapeutic efficacy and prognosis of pancreatic cancer.

The article "miR-193a-5p Enhances the Radioresistance of Pancreatic Cancer Cells by Targeting ZFP57 and Activating the Wnt Pathway" was published in 2022. Journal: J Oncol.

ZFP57, a member of KRAB-ZFPs (KRAB zinc finger family of proteins), interacts with DNMT1 (DNA methyltransferase 1) and regulates DNA methylation level [4]. Abnormal DNA methylation is closely associated with oncogenesis [5]. ZFP57 can inactivate the Wnt/*β*-catenin pathway and inhibit cancer cell proliferation [6]. The Wnt/*β*-catenin pathway is a conservative signaling axis involved in various physiological processes (e.g., proliferation, differentiation, apoptosis, migration, invasion, and tissue balance). It has been shown that the dysregulation of the Wnt/*β*-catenin signaling promotes the occurrence and development of various cancers by regulating the EGFR (epidermal growth factor receptor), Hippo/YAP, and NF-*κ*B (nuclear kappa-B) pathways [7–9]. In addition to the close connections between the Wnt pathway and human cancer initiation and growth, Wnt pathway also involves in chemotherapy resistance of cancers by regulating DNA damage repair [10, 11]. Accumulating evidence has recently shown that miRNAs enhance radioresistance of tumors by regulating specific target genes and activating the Wnt/*β*-catenin pathway [12].

miRNAs (microRNAs) are a class of small noncoding RNAs involved in cell proliferation, apoptosis, and differentiation. Many recent studies have shown that miRNAs participate in cellular processes and have close connections with the occurrence and development of tumors [13, 14]. Large differences have been observed in miRNA expression profiles of pancreatic cancer tissues and the paired cancerous tissues, hence suggesting the potential roles of miRNAs in pancreatic cancer [15]. miRNAs have been found related to the regulation of pancreatic cancer radiosensitivity via affecting DNA damage, cell apoptosis, or cell cycle alteration [16]. However, whether miR-193a-5p could influence the radioresistance of PCC (pancreatic cancer cells) is diminished.

In our study, ZFP57 was downregulated in pancreatic cancer after radiotherapy and the Wnt/*β*-catenin pathway was activated, thereby enhancing the radioresistance of pancreatic cancer cells. miR-193a-5p was predicted as the upstream regulator of ZFP57 by bioinformatics. Further, we investigated the role of the miR-193a-5p/ZFP57/Wnt pathway in radioresistance. Our findings may supply new clues for the treatment of pancreatic cancer.

The article "miR-193a-5p Enhances the Radioresistance of Pancreatic Cancer Cells by Targeting ZFP57 and Activating the Wnt Pathway" was published in 2022. Journal: J Oncol.

## 2. Materials and Methods

### 2.1. Collection of Pancreatic Tumor Tissues

This study included thirty patients diagnosed with pancreatic cancer and hospitalized at Haikou People's Hospital between May 2017 and June 2020, and a RSI model was used [17]. The patients (10 males and 10 females) were divided into two groups, namely, CR+PR (complete remission and partial remission) group (*n* = 10) and SD+PD (stable disease and progressive disease) group (*n* = 10). Patients in the CR+PR group had local residual lesions within three months but no locally recurrent lesions at 12 months after radiotherapy. Patients in the SD+PD group had incomplete recession of primary cancers or metastases for over three months and local recurrence of primary cancers or metastases within 12 months after radiotherapy. This study has been approved by the Ethics Committee of Haikou People's Hospital. All study participants provided written informed consent before participating in the study.

### 2.2. Cell Culture

BxPC-3 human PCC purchased from the Shanghai Cell Bank of Chinese Academy of Sciences were cultured in the Roswell Park Memorial Institute 1640 (RPMI 1640) medium (Genom, Zhejiang, China) containing 5% fetal bovine serum. The cells were incubated at 5% CO_2_ at 37°C, with one passage every three days. When the BxPC-3 cells reached about 85% density, they were digested with an appropriate amount of trypsin (Genom, Zhejiang, China) and resuspended. Then, the cells were inoculated to the 96-well plate (Corning, Corning, NY, USA) at a concentration of 3 × 10^5^ cells per well and cultured conventionally for 12 h.

### 2.3. Cell Irradiation and Culture of Irradiation-Resistant Cells

Siemens Primus Linear Accelerator (Siemens, Germany) was used to generate a 6 MV X-ray beam for radiotherapy at a radiation dose rate of 3 Gy per minute. The X-ray beam was delivered vertically at 0, 2, 4, 6, and 8 Gy, respectively. The radiation field was 10 cm × 10 cm, with a source-to-target distance of 3 cm. The survival fraction was estimated after irradiation. According to the literature [18], when the parental BxPC-3 cells (named BxPC-3-P) entered the logarithmic growth phase (70%-80%), X-ray beam was generated with a linear accelerator for the radiotherapy. The culture medium was replaced after 24 h of irradiation. When the cells continued to grow or new colonies were formed, the cells were digested and loaded into another flask. The cells which reached 70-80% confluency were reirradiated at 4 Gy for a total dose of 40 Gy. The cells obtained after the above procedures were screened out and identified as radioresistant pancreatic cancer cells BxPC-3-RR^12^.

The article "miR-193a-5p Enhances the Radioresistance of Pancreatic Cancer Cells by Targeting ZFP57 and Activating the Wnt Pathway" was published in 2022. Journal: J Oncol.

### 2.4. Cell Transfection and Grouping

Into a 6-well plate, the BxPC-3 cells were inoculated at an appropriate concentration and cultured for twenty-four hours. The cells were then harvested for transfection according to the manual (article no.: 11668030, Thermo Fisher Scientific, Waltham, MA, USA). All of the lentiviral vectors used were designed by Guangzhou FulenGen Co., Ltd. The cells were randomly divided into the following groups: BxPC-3-P (parental BxPC-3 PCC), BxPC-3-RR (radioresistant PCC subtype), IR^−^+BxPC-3-P (BxPC-3-P cells exposed to 2 Gy IR^−^), IR^−^+BxPC-3-RR (BxPC-3-RR cells exposed to 2 Gy IR^−^), IR^+^+BxPC-3-P (BxPC-3-P cells exposed to 2 Gy IR^+^), IR^+^+BxPC-3-RR (BxPC-3-RR cells exposed to 2 Gy IR^+^), sh-NC (BxPC-3-P cells containing empty vectors), sh-ZFP57-1 (BxPC-3-P cells containing sh-ZFP57-1), sh-ZFP57-2 (BxPC-3-P cells containing sh-ZFP57-2), IR^−^+sh-NC (BxPC-3-P cells containing 2 Gy IR^−^), IR^−^+sh-ZFP57-2 (BxPC-3-P cells containing sh-ZFP57-2 and exposed to 2 Gy IR^−^), IR^+^+sh-NC (BxPC-3-P cells containing sh-NC and exposed to 2 Gy IR^+^), IR^+^+ZFP57-2 (BxPC-3-P cells containing ZFP57-2 and exposed to 2 Gy IR^+^), vector (BxPC-3-RR cells containing pc DNA 3.0 empty vectors), ZFP57 (BxPC-3-P cells containing pc DNA 3.0 ZFP570), IR^−^+vector (vectors exposed to 2 Gy IR^−^), IR^−^+ZFP57 (ZFP572 cells exposed to Gy IR^−^), IR^+^+vector (vectors exposed to 2 Gy IR^+^), IR^+^+ZFP57 (ZFP57 exposed to 2 Gy IR^+^), NC mimic+vector (BxPC-3-RR cells containing NC mimics and ZFP control), NC mimic+ZFP57 MUT (BxPC-3-RR cells containing NC mimics and ZFP57 MUT), miR-193a-5p mimic+vector (BxPC-3-RR cells containing ZFP control and miR-193a-5p mimics), and miR-193a-5p mimic+ZFP57 MUT (BxPC-3-RR cells containing ZFP57 MUT and miR-193a-5p mimics). The cells at forty-eight hours after transfection were collected for subsequent use^12^.

### 2.5. Total RNA Extraction and RT-qPCR

Total RNA was extracted from the cells using the TRIzol reagent (Invitrogen, Carlsbad, CA, USA) according to the instruction manual. The extracted RNA was reversely transcribed into cDNA using the PrimeScript RT Reagent Kit (TaKaRa, Dalian, China). cDNA amplification and quantification were carried out using SYBR Green mix (TaKaRa, Dalian, China) on the Applied Biosystems 7500 instrument (Thermo Fisher Scientific, Waltham, MA, USA). The primer sequences are shown in Table 1. Using the 2^-*ΔΔ*Ct^ method, the relative expression of genes was calculated^9^.

### 2.6. Colony Formation Assay

The BxPC-3 cells in different groups were exposed to 0, 2, 4, 6, and 8 Gy radiotherapy, respectively, followed by cell culture for forty-eight hours. After changing the medium, BxPC-3 cells were further cultured until colony formation. After phosphate buffer (Thermo Fisher Scientific, Waltham, MA, USA) washing, the cells were fixed in an appropriate amount of methanol for 20 minutes. We counted the number of colonies containing ≥50 cells after they were stained with crystal violet (0.2%) for 10 minutes. Colony formation rate (%) = (number of colonies/number of inoculated cells) × 100%; survival fraction (SF2) = colony formation rate of the experimental group/colony formation rate of the control group; radiotherapy sensitization ratio = survival fraction before silencing/survival fraction after silencing.

The article "miR-193a-5p Enhances the Radioresistance of Pancreatic Cancer Cells by Targeting ZFP57 and Activating the Wnt Pathway" was published in 2022. Journal: J Oncol.

### 2.7. Cell Counting Kit-8 (CCK-8) Assay

We assessed cell viability using CCK-8 assay (CCK-8; Beyotime, Shanghai, China). Into 96-well plates, the cells (5,000 cells per well) in each group were inoculated, followed by incubation for 48 h. Next, 10 *μ*l of CCK-8 solution was added per well to incubate the cells for one hour. Using the Bio-Rad Microplate Reader (Bio-Rad, Hercules, CA, USA), the absorbance was detected at a wavelength of 450 nm.

### 2.8. Western Blotting

Radioimmunoprecipitation assay (RIPA) lysis buffer (Beyotime, Shanghai, China) with protease inhibitor cocktail (Sigma, St. Louis, MO, USA) was added and mixed properly. The cells were centrifuged at 13,000 rpm for 10 min after lysis on ice for half an hour, and the supernatant was collected. Bicinchoninic acid (BCA) (Pierce, Rockford, IL, USA) was added for quantification of the total protein. The 10% sodium dodecyl sulphate-polyacrylamide gel electrophoresis (SDS-PAGE) gel was prepared for electrophoresis, and the separated proteins were transferred onto polyvinylidene fluoride (PVDF) membranes, which were then sealed with defatted milk (5%) prepared with tris buffered saline-tween (TBST) (Thermo Fisher Scientific, China) and shaken on a shaker for 1 h. The membrane was incubated with the following primary antibodies at 4°C overnight: Cyclin D1 (1 : 200, ab16663, Abcam, Cambridge, MA, USA), Cdk4 (1 : 1,000, ab108357, Abcam, Cambridge, MA, USA), Bax (1 : 1,000; ab32503, Abcam, Cambridge, MA, USA), Cleaved Caspase-3 (1 : 5,000/500; ab214430-mouse, ab32042-human, Abcam, Cambridge, MA, USA), c-Myc (1 : 1,000; ab32072, Abcam, Cambridge, MA, USA), Bcl-2 (1 : 1,000; ab194583, Abcam, Cambridge, MA, USA), *γ*-H2AX (1 : 5,000; ab81299, Abcam, Cambridge, MA, USA), *β*-catenin (1 : 5,000; ab3257, Abcam, Cambridge, MA, USA), and Ki67 (1 : 5,000; ab231172, Abcam, Cambridge, MA, USA). The membrane was washed with TBST (three times, 5 min each time) and incubated with the peroxidase-labeled IgG secondary antibody (1 : 2,000, ab205718, Abcam, Cambridge, MA, USA) for one hour. Finally, the protein bands were visualized using the enhanced electrochemiluminescence (ECL) chemiluminescent substrate (Pierce, Rockford, IL, USA). GAPDH (1 : 2500, ab9485, Abcam, Cambridge, MA, USA) was used as an internal reference^6^.

The article "miR-193a-5p Enhances the Radioresistance of Pancreatic Cancer Cells by Targeting ZFP57 and Activating the Wnt Pathway" was published in 2022. Journal: J Oncol.

### 2.9. Nude Mouse Experiment

Sixty female BALB/c nude mice at 3-7 weeks of age were purchased from Guangdong Animal Medicine Center. The animals were randomly grouped using a random number table: IR^−^+vector (vectors exposed to 10 Gy IR^−^), IR^−^+ZFP57 (ZFP57 exposed to 10 Gy IR^−^), IR^+^+vector (vectors exposed to Gy IR^+^), and IR^+^+ZFP57 (ZFP57 exposed to 10 Gy IR^+^), with 5 mice in each group. All animals were bred in a laminar flow hood. The BxPC-3-RR cells with ZFP57 overexpression or transfected with the corresponding control were resuspended in the DMEM high-glucose medium (Thermo Fisher Scientific, Waltham, MA, USA). The density of the cell suspension was adjusted to 3 × 10^5^/ml. Then, 0.2 ml of the suspended pancreatic cancer cells was injected subcutaneously into the animals (the right lower limb). The formed tumor was exposed to 10 Gy radiotherapy. The mice were bred as before and exposed to irradiation every two days for three times consecutively. This cycle was repeated three times before the subsequent experiments. At four weeks after the injection, several mice were killed every week. We harvested and weighed the tumors and measured the volume. Every procedure was approved by the Animal Care and Use Committee of Haikou People's Hospital.

### 2.10. RNA Pull-Down Assay

miR-193a-5p and the reference RNA were labeled with the 3′ End Biotinylation Kit (Thermo, Waltham, MA, USA). A biotin-labeled RNA pull-down assay was conducted to determine the miRNA-protein interaction (Thermo, Waltham, MA, USA). The biotin-labeled RNA and the streptavidin beads were mixed in the RNA capture buffer at room temperature for half an hour. The cell lysates were collected and mixed with the miR-193a-5p-bound magnetic beads at four centigrade degree on a rotator for 1 h. The magnetic beads were fully washed. RNA was recovered from the magnetic beads, and RT-qPCR was performed.

### 2.11. Dual-Luciferase Reporter Gene Assay

MT (mutant) or WT (wild-type) ZFP57 fragment which covered the binding site of miR-193a-5p was inserted into pGL3-basic vectors (provided by Promega, Madison, WI, USA). The BxPC-3 cells were added with miR-193a-5p mimics or the corresponding NC for luciferase determination. Forty-eight hours later, the luciferase activity was assessed by the luciferase reporter system (Promega, Madison, WI, USA).

The article "miR-193a-5p Enhances the Radioresistance of Pancreatic Cancer Cells by Targeting ZFP57 and Activating the Wnt Pathway" was published in 2022. Journal: J Oncol.

### 2.12. Statistical Analysis

GraphPad Prism 8.0.1 (GraphPad Software Inc., San Diego, CA, USA) was utilized. The data were described as mean ± standard deviation (SD) of 3 independent experiments. An independent sample *t*-test or one-way ANOVA was used if appropriate. Tukey's post hoc analysis was performed. Two-sided *P* < 0.05 indicated significant difference.

## 3. Results

### 3.1. ZFP57 Was Downregulated in Radioresistant Pancreatic Cancer Cells

Ten pancreatic cancer cases achieving CR+PR and ten cases achieving SD+PD were recruited from our hospital. RT-qPCR was performed to determine the mRNA level of ZFP57 in tissues of each group. The results showed that before and after radiotherapy, the mRNA level of ZFP57 in cases achieving CR+PR was significantly higher than that in cases achieving SD+PD. The mRNA level of ZFP57 in the SD+PD group decreased noticeably after radiotherapy (Figure 1(a)). Later, the ZFP57 protein level in tissues of each group was determined by WB, and a similar trend was found as PCR (Figure 1(b)). PAAD data were downloaded from the TCGA database, and the survival curve was plotted. The results showed that the survival rate of cases with high ZFP57 expression in either group was much higher compared to cases with low ZFP57 expression (Figure 1(c)). Hence, the ZFP57 expression might be related to the prognosis of pancreatic cancer. Further, the radioresistant pancreatic cancer cell subtype BxPC3-RR was built by repeated irradiation of the BxPC3 cells. Our purpose was to validate the role of ZFP57 in radioresistance on the cellular level. The colony formation assay indicated that the parental BxPC3-P cells and the resistant cell subtype BxPC3-RR had a lower survival fraction after exposed to 2, 4, and 8 Gy IR. Moreover, a dose-dependent relationship was observed. Besides, the survival fraction of BxPC3-P cells was significantly lower than that of its subtype BxPC3-RR (Figure 1(d)). We also investigated the protein and mRNA expressions of ZFP57 in the parental BxPC3-P cells and its subtype BxPC3-RR cells under different doses of radiotherapy (IR^+^ and IR^−^). RT-qPCR and WB results showed that under different irradiation doses (IR^+^ and IR^−^), the protein and mRNA expressions of ZFP57 in the parental BxPC3-P cells were higher compared to the BxPC3-RR cells (Figures 1(e) and 1(f)). The results above suggested that the ZFP57 expression might be related to the radioresistance of pancreatic cancer. A high ZFP57 expression was associated with a higher survival rate. In the CR+PR group, the ZFP57 expression of PCC was significantly higher than that in the SD+PD group. Besides, ZFP57 expression in PCC was downregulated by radiotherapy.

The article "miR-193a-5p Enhances the Radioresistance of Pancreatic Cancer Cells by Targeting ZFP57 and Activating the Wnt Pathway" was published in 2022. Journal: J Oncol.

### 3.2. Inhibiting ZFP57 Ameliorated the Radiosensitivity of PCC

As found above, ZFP57 was downregulated in radioresistant PCC. Besides, the radioresistant cells had a higher survival fraction than the parental BxPC3-P cells. The BxPC3-P cells were further transfected with shRNA to inhibit ZFP57 expression. Our purpose was to verify the viability of BxPC3-P cells with low ZFP57 expression. The ZFP57 expression was downregulated significantly after transfection with two different plasmids, while the decrease was greater after transfection with sh-ZFP57-2 (Figure 2(a)). Later, the survival fractions of BxPC3-P cells containing sh-NC or sh-ZFP-2 and exposed to different irradiation doses (IR^+^ and IR^−^) were estimated, and it was found that the survival fractions of BxPC3-P cells which were transfected with sh-ZFP-2 were significantly higher compared to those transfected with sh-NC (Figure 2(b)). The MTT assay showed that the BxPC3-P cell viability was higher after transfection with sh-ZFP-2 under different irradiation doses. Besides, exposure to IR^+^ had a greater effect on the viability of BxPC3-P cells than IR^−^ (Figure 2(c)). The above results indicated that inhibiting ZFP57 ameliorated the radiosensitivity of pancreatic cancer cells. According to WB results, compared to the BxPC3-P cells transfected with sh-NC, the cyclin D1 and CDK4 expressions were upregulated after transfection with sh-ZFP-2 and exposure to irradiation. Meanwhile, the Bax and cleaved caspase-3 expressions were downregulated, Bcl-2 expression was upregulated, and the *γ*-H2AX expression was downregulated (Figure 2(d)). The expressions of *β*-catenin and c-Myc, which were involved in the Wnt/*β*-catenin pathway, were downregulated (Figure 2(e)). The results above indicated that inhibiting ZFP57 ameliorated the radiosensitivity of pancreatic cancer cells, the viability of which was inhibited via the Wnt/*β*-catenin pathway. As a result, malignant progression of PCC was promoted, and the radioresistance of PCC was enhanced.

### 3.3. ZFP57 Overexpression Ameliorated Radioresistance of PCC

Based on our preliminary experiments, it was found that the ZFP57 expression could influence PCC proliferation and viability via the Wnt/*β*-catenin pathway. As a result, the radiosensitivity of PCC was ameliorated. Besides, we further verified the proliferation of radioresistant PCC subtype BxPC3-RR with ZFP57 overexpression. Our purpose was to investigate the role of ZFP57 expression in the radioresistance of PCC. ZFP57 overexpression in BxPC3-RR cells was induced by transfection with the pc DNA 3.0 plasmid. The transfection efficiency is available in Figure 3(a). Compared with the empty plasmid, the ZFP57 expression was upregulated in BxPC3-RR cells transfected with pc DNA 3.0 ZFP57. Next, we detected the survival fractions of BxPC3-RR cells transfected with the empty plasmid and pc DNA 3.0 ZFP57 and exposed to different irradiation doses (IR^+^ and IR^−^). It was found that the survival fractions of the BxPC3-RR cells transfected with pc DNA 3.0 ZFP57 under all irradiation doses were reduced compared to cells transfected with empty plasmids (Figure 3(b)). As shown by the results of CCK-8 assay, under different irradiation doses, transfection with pc DNA 3.0 ZFP57 resulted in higher viability of BxPC3-RR cells. Besides, the irradiation dose IR^+^ had a greater effect on BxPC3-P cell viability than IR^−^ (Figure 2(c)). The WB results showed that the expressions of cyclin D1 and CDK4 were downregulated in the BxPC3-RR cells transfected with pc DNA 3.0 ZFP57 and exposed to the irradiation, compared with the BxPC3-RR cells transfected with the empty plasmid. The expressions of cleaved caspase-3 and Bax were downregulated, similar to Bcl-2. However, the expression of *γ*-H2AX was upregulated (Figure 2(d)). The expressions of c-Myc and *β*-catenin, which were related to the Wnt/*β*-catenin pathway, were upregulated (Figure 2(e)). The above results indicated that inhibiting ZFP57 ameliorated the radioresistance of PCC. Moreover, the proliferation of PCC was decreased by acting on the Wnt/*β*-catenin pathway. Consequently, the malignant progression of PCC was promoted, and the radioresistance of PCC was enhanced.

The article "miR-193a-5p Enhances the Radioresistance of Pancreatic Cancer Cells by Targeting ZFP57 and Activating the Wnt Pathway" was published in 2022. Journal: J Oncol.

### 3.4. ZFP57 Overexpression Suppressed the Growth of Transplanted Tumor in Irradiated Mice

A nude mouse model of radioresistant pancreatic cancer was constructed by injecting BxPC3-RR cells with ZFP5 overexpression into the nude mice. Four weeks later, the tumor samples were collected after killing the mice. The dissected transplanted tumors are shown in Figure 4(a). The tumor size increased over time. The tumors with ZFP57 overexpression shrank in size significantly compared to the control group (Figure 4(b)). The former also had a considerable decrease in weight than the latter (Figure 4(c)). The WB assay showed that the expressions of relevant proteins in mice with ZFP57-overexpressing pancreatic cancer were increased compared to the control group. Specifically, ZFP57 overexpression downregulated Ki67 and CDK4 and upregulated Bax and *γ*-H2AX. Moreover, the *β*-catenin protein was downregulated (Figure 4(d)). The above results showed that ZFP57 overexpression inhibited the transplanted tumor growth in mice with radioresistant pancreatic cancer by regulating the expressions of relevant proteins.

### 3.5. ZFP57 Ameliorated Radioresistance of PCC by Inhibiting the Wnt Pathway

Based on the preliminary *in vivo* and *in vitro* experiments, it was found that ZFP57 affected the expressions of *β*-catenin and *γ*-H2AX, proteins involved in the Wnt/*β*-catenin pathway. The use of Wnt/*β*-catenin pathway agonist SKL2001 on the Wnt/*β*-catenin pathway or the potential role of ZFP57 overexpression in BxPC3-RR cells was determined on the cellular level. The colony formation assay suggested that the survival fraction of cancer cells in each group decreased with the treatment of irradiation, which was dose-dependent. Besides, the BxPC3-RR cells with ZFP57 overexpression had a significantly lower survival fraction regardless of the use of SKL2001 (Figure 5(a)). The cell viability as detected by CCK-8 showed a similar trend (Figure 5(b)). The Wnt/*β*-catenin pathway agonist SKL2001 partially counteracted the effect of ZFP57 on the proliferation of BxPC3-RR cells exposed to irradiation. The expressions of relevant proteins were further determined by WB. The results showed that ZFP57 overexpression downregulated cyclin D1, CDK4, and Bcl-2 and upregulated Bax and *γ*-H2AX. Moreover, c-myc and *β*-catenin were downregulated in ZFP57 overexpressed cells. The above results suggested that ZFP57 might inhibit the WNT pathway in PCC, thereby ameliorating radioresistance.

The article "miR-193a-5p Enhances the Radioresistance of Pancreatic Cancer Cells by Targeting ZFP57 and Activating the Wnt Pathway" was published in 2022. Journal: J Oncol.

### 3.6. miR-193a-5p Targeted ZFP57 and Suppressed ZFP57 Expression

To investigate the role of miRNAs in the radioresistance of PCC, upregulated genes (GEO accession number GSE104965) were identified from the miRWalk database (http://mirwalk.umm.uni-heidelberg.de/) and GEO database. miRNAs which may regulate ZFP57 were analyzed. Seven miRNAs were screened out, namely, miR-675-5p, miR-193a-5p, miR-675-5p, miR-744-5p, miR-502-3p, miR-193a-3p, miR-149-5p, and miR-616-3p (Figure 6(a)). The binding of ZFP57 and miR-193a-5p was evaluated by RNA pull-down assay (Figure 6(b)). The dual-luciferase reporter assay showed that after transfection of BxPC3-RR cells with miR-193a-5p mimics, the fluorescence intensity decreased significantly in the ZFP57-WT 3′UTR group. However, there was no significant difference in the ZFP57-MUT 3′UTR group (Figure 6(c)). This result indicated miR-193a-5p targeted ZFP57 in BxPC3-RR cells. Next, miR-193a-5p expression was inhibited or enhanced by transfecting BxPC3-RR cells with miR-193a-5p inhibitors or mimics. The ZFP57 expression was detected using WB and RT-qPCR, and it was revealed that miR-193a-5p inhibition in BxPC3-RR cells increased the protein and mRNA levels of ZFP57 significantly (Figure 6(d)). On the contrary, overexpression of miR-193a-5p in BxPC3-RR cells caused a noticeable decrease in the mRNA and protein expressions of ZFP57 (Figure 6(e)). To determine dynamic changes of miR-193a-5p expression before and after radiotherapy in radioresistant pancreatic cancer, RT-qPCR was carried out to determine miR-193a-5p levels before and after radiotherapy in tumor samples collected from cases responsive and unresponsive to radiotherapy. The miR-193a-5p level in PCC collected from unresponsive cases was consistently higher than that from responsive cases. Besides, the miR-193a-5p level in PCC from unresponsive cases was significantly higher after irradiation than before (Figure 6(f)). Similarly, in *in vitro* experiments, the miR-193a-5p level in BxPC3-RR cells was significantly increased compared to BxPC3-P cells (Figure 6(g)). The above results suggested that miR-193a-5p was highly expressed in radioresistant PCC and miR-193a-5p might increase the radioresistance of PCC via targeting ZFP57.

The article "miR-193a-5p Enhances the Radioresistance of Pancreatic Cancer Cells by Targeting ZFP57 and Activating the Wnt Pathway" was published in 2022. Journal: J Oncol.

### 3.7. The Inhibitory Role of ZFP57 in Postirradiation Viability of PCC Was Partially Reversed by miR-193a-5p Overexpression

The effect of miR-193a-5p overexpression on the proliferation of irradiated BxPC3-RR cells with ZFP57 (mut) overexpression was investigated. It was found that the survival fraction of cells declined in an IR dose-dependent manner. The mutation resulted in the loss of targeting potential of ZFP57 by miR-193a-5p but contained the function of ZFP57. Transfection of miR-193a-5p mimics into cells with ZFP57 (mut) overexpression reduced the survival fraction compared to BxPC3-RR cells which were transfected with miR-193a-5p mimics (Figure 7(a)). Moreover, the cell viability as detected by the MTT assay showed a similar trend (Figure 7(b)). The expressions of relevant proteins were determined by WB assay. CDk4 and Cyclin D1 (cell cycle-related proteins) and Bcl-2 (the apoptosis-related protein) were downregulated in ZFP57 (mut) overexpressed cells. The upregulation of proteins induced by miR-193a-5p mimics was reversed by ZFP57 (mut) overexpression. Cleaved caspase-3 and Bax (apoptosis-related protein) and *γ*-H2AX (DNA repair-related protein) were upregulated after ZFP57 (mut) overexpression. The downregulation of proteins induced by miR-193a-5p overexpression was further promoted after ZFP57 (mut) overexpression (Figure 7(c)). Similarly, the expressions of c-Myc and *β*-catenin proteins related to the Wnt/*β*-catenin pathway were decreased after ZFP57 (mut) overexpression. On the contrary, the upregulation of proteins induced by increased miR-193a-5p expression was reversed by ZFP57 (mut) (Figure 7(d)). Taken together, overexpressed miR-193a-5p partially reversed the inhibitory effect of ZFP57 MUT on pancreatic cancer cell proliferation after irradiation. Moreover, this effect was achieved by the regulation of the Wnt/*β*-catenin pathway.

The article "miR-193a-5p Enhances the Radioresistance of Pancreatic Cancer Cells by Targeting ZFP57 and Activating the Wnt Pathway" was published in 2022. Journal: J Oncol.

## 4. Discussion

Pancreatic cancer is a common malignancy of the digestive tract and is generally known for its very poor prognosis^1^. Recently, a growing number of signaling pathways and molecules have been proven to participate in the occurrence and development of pancreatic cancer. The Wnt/*β*-catenin pathway is involved in the regeneration, proliferation, and differentiation of cancer stem cells, which plays a vital role in tumor treatment. Radiotherapy, together with chemotherapy, is an essential treatment for pancreatic cancer, especially for cases with locally advanced cancer, as it can dramatically improve the survival rate [19]. However, radioresistance is a restricting factor in radiotherapy for pancreatic cancer. Enhancing radiosensitivity can improve the therapeutic effect of pancreatic cancer. miRNAs are closely related to the radiosensitivity of PCC and may be targeted for tumor diagnosis and treatment.

miRNAs participate in cell apoptosis, differentiation, and individual development. miR-193a-5p activates the AKT-mTOR pathway and promotes colorectal cancer progression [20]. Plasma miR-193a-5p may be a marker for the prognosis of colorectal cancer [21]. In recent years, it has been shown that miRNAs are involved in regulation of downstream target genes, thereby affecting radiosensitivity. In radioresistant esophageal squamous cell cancer cells, circRNA_100367 bound to miR-217 and regulated Wnt3 expression, thereby affecting radioresistance [22]. In glioblastoma, the Wnt/*β*-catenin pathway was activated by miR-301a overexpression, and radioresistance was promoted [12]. According to the literature, miR-193a-5p is related to the radiosensitivity of breast cancer cells by promoting cell apoptosis while inhibiting cell proliferation [23]. The existing studies have proven the important roles of miRNAs in cancer treatment, which provide clues for enhancing the radiosensitivity of cancers.

Transcription factor ZFP57 was first identified as an undifferentiated cell-specific gene in F9 embryonic carcinoma cells. A large number of reports have been published regarding the role of ZFP57 in tumor cell proliferation [24, 25]. One study showed that ZFP57 was downregulated in breast cancer, while ZFP57 overexpression inhibited breast cancer cell proliferation by inhibiting the Wnt/*β*-catenin pathway [6]. However, there are few reports on the role of ZFP57 in radioresistance of cancers. Of note, the WNT/*β*-catenin pathway is a highly conservative and strictly controlled molecular mechanism. This pathway regulates embryonic development and cell proliferation and differentiation and plays an important role in oncogenesis and development of hepatocellular carcinoma and cholangiocarcinoma [26], which may be a candidate target for antitumor treatment [27, 28]. Its role in promoting DNA damage repair and inhibiting cell apoptosis may be related to radioresistance of cancers [29].

The article "miR-193a-5p Enhances the Radioresistance of Pancreatic Cancer Cells by Targeting ZFP57 and Activating the Wnt Pathway" was published in 2022. Journal: J Oncol.

## 5. Conclusion

In this study, we found that ZFP57 expression in radioresistant PCC was low but the level of miR-193a-5p was high. Overexpressed miR-193a-5p targeted ZFP57 and inhibited ZFP57 expression, thereby suppressing the activation of the Wnt pathway and enhancing the radioresistance of PCC. Taken together, miR-193a-5p targeted ZFP57 and inhibited ZFP57 expression, thereby activating the Wnt/*β*-catenin pathway and enhancing the radioresistance of PCC.

## Figures and Tables

**Figure 1:** The correlation between ZFP57 expression and radioresistance of PCC was assessed. 10 pancreatic cancer cases achieving CR+PR and 10 patients achieving SD+PD were recruited. Cancerous tissues from these cases were exposed to X-ray irradiation. (a) ZFP57 expression in tissues of pancreatic cancer before irradiation as detected by RT-qPCR. (b) ZFP57 expression in pancreatic cancer tissues before irradiation as detected by WB. (c) Survival curve of TCGA PAAD cases achieving CR+PR and SD+PD after radiotherapy based on ZFP57 expression. BxPC3 cells (specifically named parental BxPC3-P cells in the present study) were exposed to repeated X-ray irradiations to induce the radioresistant cell subtype BxPC3-RR. (d) Survival fractions of BxPC3-P and BxPC3-RR cells after exposed to 0, 2, 4, and 8 Gy IR^+^ and IR^−^ as detected by the colony formation assay. (e) ZFP57 expressions in BxPC3-P and BxPC3-RR cells after exposed to 8 Gy IR^+^ and IR^−^ as detected by qPCR. (f) ZFP57 expression in BxPC3-P and BxPC3-RR cells after exposed to 8 Gy IR^+^ and IR^−^ as detected by WB. ^∗∗∗^*P* < 0.001 and ^∗∗^*P* < 0.01.

**Figure 2:** The radiosensitivity of BxPC3-P cells with induced ZFP57 overexpression was evaluated. (a) The ZFP57 expression was inhibited by lentiviral transfection. The ZFP57 expression was determined in BxPC3-P cells transfected with sh-ZFP57-1, sh-ZFP57-2, and the corresponding control by qPCR. After exposure of the BxPC3-P cells transfected with sh-ZFP57-2 and the corresponding control to 8 Gy irradiation, (b) the survival fraction estimated by colony formation assay. (c) Cell viability revealed by CCK-8 assay. (d) The expressions of the cell cycle-related proteins cyclin D1 and CDK4; apoptosis-related proteins Bax, Bcl-2, and cleaved caspase-3; and DNA repair-related protein *γ*-H2AX revealed by WB assay. (e) The expressions of *β*-catenin and c-Myc revealed by WB assay. ^∗∗∗^*P* < 0.001 and ^∗∗^*P* < 0.01.

The article "miR-193a-5p Enhances the Radioresistance of Pancreatic Cancer Cells by Targeting ZFP57 and Activating the Wnt Pathway" was published in 2022. Journal: J Oncol.

**Figure 3:** The radiosensitivity of BxPC3-RR cells with induced ZFP57 overexpression was evaluated by detecting cancer cell proliferation and viability after transfection with pc DNA 3.0 and exposure to different irradiation doses. (a) The ZFP57 expression was determined in BxPC3-RR cells transfected with pc DNA 3.0 ZFP57 and the corresponding control. The BxPC3-P cells transfected with sh-ZFP57-2 and the corresponding control were exposed to 8 Gy irradiation. Then, (b) the survival fraction of the BxPC3-RR cells was estimated by colony formation assay. (c) CCK-8 assay was performed to assess the BxPC3-RR cell viability. (d) WB assay was performed to determine the expressions of cyclin D1 and CDK4 (cell cycle-related proteins); Bax, Bcl-2, and cleaved caspase-3 (apoptosis-related proteins); *γ*-H2AX (DNA repair-related protein); and (e) *β*-catenin and c-Myc expressions. ^∗∗∗^*P* < 0.001, ^∗∗^*P* < 0.01, and ^∗^*P* < 0.05.

**Figure 4:** The BxPC3-RR cells with ZFP57 overexpression and transfected with the corresponding control were injected into subcutaneous tissues of nude mice. Then, the transplanted tumor was irradiated by 10 Gy of different types of radiation once every two days for three times consecutively. (a) The nude mice with the transplanted tumors were killed after four weeks of radiotherapy at 10 Gy, and the photos were taken at the transplanted tumors. (b) The transplanted tumor volume was measured every week after radiotherapy at 10 Gy. (c) The weight of the transplanted tumor was determined. (d) The expressions of ZFP57, Ki67, Bax, CDK4, *β*-catenin, and *γ*-H2AX were determined in the transplanted tumors by WB. ^∗∗∗^*P* < 0.001 and ^∗∗^*P* < 0.01.

**Figure 5:** To verify how the regulatory effect of ZFP57 on the WNT pathway affected radiosensitivity of PCC, ZFP57 overexpression was induced in BxPC3-RR cells with or without the incubation of SKL2001, followed by radiotherapy. (a) Survival fraction of the BxPC3-RR cells. (b) Cell viability. (c) Expressions of CDK4 and cyclin D1 (related to cell cycle), Bax and Bcl-2 (proteins related to apoptosis), cleaved caspase-3 (a protein related to DNA repair *γ*-H2AX), and proteins involved in the WNT pathway (d) *β*-catenin and c-Myc. ^∗∗^*P* < 0.01 and ^∗^*P* < 0.05.

**Figure 6:** Upstream miRNAs regulating ZFP57 were analyzed. (a) miRWalk database was used in conjunction with the GEO database to predict miRNAs targeting ZFP57. (b) RNA pull-down assay was performed on BxPC3-RR cells. The enriched miRNA was determined by qPCR. (c) The binding site of ZFP and miR-193a-5p was predicted by bioinformatics tools. The prediction was further verified by the luciferase reporter gene assay. The dual-luciferase reporter gene assay was performed on the transfected BxPC3-RR cells. (d) In BxPC3-RR cells, miR-193a-5p expression was silenced. mRNA and protein expressions of ZFP57 were determined by qPCR and WB assay, respectively. (e) miR-193a-5p overexpression was induced in BxPC3-P cells. The protein and miRNA levels of ZFP57 were determined by WB and qPCR. (f) miR-193a-5p levels in pancreatic cancer tissues were determined by qPCR. (g) Pancreatic cancer cells were exposed to IR, and the miR-193a-5p expression was detected by qPCR subsequently. ^∗∗∗^*P* < 0.001 and ^∗∗^*P* < 0.01.

The article "miR-193a-5p Enhances the Radioresistance of Pancreatic Cancer Cells by Targeting ZFP57 and Activating the Wnt Pathway" was published in 2022. Journal: J Oncol.

**Figure 7:** (a) The survival fraction of BxPC3-RR cells detected by colony formation assay after exposure to 0, 2, 4, and 8 Gy irradiation. (b) The CCK-8 assay was conducted to determine the viability of BxPC3-RR cells after exposure to 8 Gy irradiation. (c) WB was conducted to determine the expressions of CDK4 and cyclin D1 (proteins related to cell cycle); Bax, Bcl-2, and cleaved caspase-3 (proteins related to cell apoptosis); *γ*-H2AX (a protein related to DNA repair); and *β*-catenin and c-Myc in BxPC3-RR cells after exposure to 8 Gy irradiation. ^∗∗^*P* < 0.01 and ^∗^*P* < 0.05.

**Table 1:** Sequences of PCR primers used in this study.

Gene	Sequences
GAPDH	
Forward (5′-3′)	TGTGGGCATCAATGGATTTGG
Reverse (5′-3′)	ACACCATGTATTCCGGGTCAAT
ZFP57	
Forward (5′-3′)	CAGAGGGTCCTTTACCAGGAT
Reverse (5′-3′)	CTCTCAGACTGGGATGTTGTTC
miR-193a-5p	
Forward (5′-3′)	GTCTTTGCGGGCGAG
Reverse (5′-3′)	GTCCAGTTTTTTTTTTTTTTTCATCTC
miR-744-5p	
Forward (5′-3′)	CGGGGCTAGGGCTAAC
Reverse (5′-3′)	TCCAGTTTTTTTTTTTTTTTGCTGT
miR-675-5p	
Forward (5′-3′)	GGAGAGGGCCCACA
Reverse (5′-3′)	TCCAGTTTTTTTTTTTTTTTCACTGT
miR-502-3p	
Forward (5′-3′)	AATGCACCTGGGCAAG
Reverse (5′-3′)	TCCAGTTTTTTTTTTTTTTTGAATCCT
miR-193a-3p	
Forward (5′-3′)	CAGAACTGGCCTACAAAGTC
Reverse (5′-3′)	CCAGTTTTTTTTTTTTTTTACTGGGA
miR-149-5p	
Forward (5′-3′)	GGCTCCGTGTCTTCACT
Reverse (5′-3′)	GTCCAGTTTTTTTTTTTTTTTGGGA
miR-616-3p	
Forward (5′-3′)	AGACTCAAAACCCTTCAGTGA
Reverse (5′-3′)	GGTCCAGTTTTTTTTTTTTTTTAAGTCA

## Data Availability

The datasets used and analyzed during the current study are available from the corresponding author on reasonable request.
